The article "Downregulation of hsa_circ_0001836 Induces Pyroptosis Cell Death in Glioma Cells via Epigenetically Upregulating NLRP1" was retracted in 2021. Reasons: signs of a paper mill; original data or images not available; unreliable results or conclusions; concerns about the data.

# Downregulation of hsa_circ_0001836 Induces Pyroptosis Cell Death in Glioma Cells *via* Epigenetically Upregulating NLRP1

**DOI:** 10.3389/fonc.2021.622727

**Published:** 2021-03-31

**Authors:** Yong Liu, Hao Wu, Jiangpeng Jing, Huanfa Li, Shan Dong, Qiang Meng

**Affiliations:** Department of Neurosurgery, The First Affiliated Hospital of Xi’an Jiaotong University, Xi’an, China

**Keywords:** glioma, circular RNA, pyroptosis, methylation, NLRP1

## Abstract

**Background:**

It has been shown that circular RNAs (circRNAs) play a vital role in the progression of glioma. Recently, hsa_circ_0001836 was found to be upregulated in glioma tissues, but the role of hsa_circ_0001836 in glioma remains unclear.

**Methods:**

EdU staining and flow cytometry assays were used to measure the viability and death of glioma cells. In addition, scanning electron microscopy (SEM) was used to observe the morphology of cells undergoing cell death.

**Results:**

Hsa_circ_0001836 expression was upregulated in U251MG and SHG-44 cells. In addition, hsa_circ_0001836 knockdown significantly reduced the viability and proliferation of U251MG and SHG-44 cells. Moreover, hsa_circ_0001836 knockdown markedly induced the pyroptosis of U251MG and SHG-44 cells, evidenced by the increased expressions of NLRP1, cleaved caspase 1 and GSDMD-N. Meanwhile, methylation specific PCR (MSP) results indicated that hsa_circ_0001836 knockdown epigenetically increased NLRP1 expression *via* mediating DNA demethylation of NLRP1 promoter region. Furthermore, downregulation of hsa_circ_0001836 notably induced pyroptosis and inhibited tumor growth in a mouse xenograft model of glioma.

**Conclusion:**

Collectively, hsa_circ_0001836 knockdown could induce pyroptosis cell death in glioma cells *in vitro* and *in vivo via* epigenetically upregulating NLRP1 expression. These findings suggested that hsa_circ_0001836 may serve as a potential therapeutic target for the treatment of glioma.

## Introduction

Glioma is the most common form of intracranial neoplasm, characterizing by uncontrolled-proliferation and unparalleled invasiveness (1–4). According to the World Health Organization (WHO) classification, gliomas can be categorized into grades I to IV based on malignancy and overall survival (5, 6). Among all the subtypes of gliomas, glioblastoma (GBM, grade IV) is the most aggressive type of malignant gliomas (7). Furthermore, glioma is a common primary malignant brain tumor with high morbidity and mortality (8). Although advances have been made in the treatment of gliomas, the overall survival time for patients with gliomas is less than 16 months after diagnosis (9, 10). Therefore, it is necessary to further investigate the pathogenesis of glioma and identify novel potential targets.

Circular RNAs (circRNAs) are a group of non-coding RNAs with a covalently closed loop structure without 5′ cap and a 3’ poly(A) tail, generated by alternative back-splicing from linear mRNA (11). Evidences have shown that circRNAs play crucial important in regulating tumor progression (12). Moreover, circRNAs can function as oncogenes or tumor suppressors in glioma progression (12, 13). Bian et al. found that circular RNA complement factor H promoted the proliferation of glioma cells through mediating miR-149/AKT1 axis (14). Wang et al. demonstrated that hsa_circ_0008225 suppressed the migration and invasion of glioma cells through sponging miR-890 (15). Recently, Qiao et al. found that hsa_circ_0001836 expression was upregulated in glioma tissues (16). However, the role and the regulatory mechanism of hsa_circ_0001836 in glioma remain largely unclear.

Thus, in this study, we aimed to explore the function of hsa_circ_0001836 in the tumorigenesis of glioma, thus providing new insights in the treatment of glioma in humans.

## Materials and Methods

### Cell Culture and Transfection

Human cortical astrocytes cell line HA1800, human glioma cell lines (U251MG, U87MG and SHG-44) were obtained from Type Culture Collection of the Chinese Academy of Sciences (Shanghai, China). Cells were maintained in DMEM (Thermo Fisher Scientific) containing 10% FBS and incubated at 5% CO_2_ at 37°C.

Negative control siRNA (siRNA-ctrl, 5’-GCGAGGCTTGACACGTATT-3’), hsa_circ_0001836 siRNA1 (5’-GATGGGGGTGGAGAAGATA-3’), hsa_circ_0001836 siRNA2 (5’-ATGGGGGTGGAGAAGATAAAT-3’), hsa_circ_0001836 siRNA3 (5’-GATGGTTGTCAATGCTATG-3’), NLRP1 siRNA1 (5’-GCTGAAGGAGTTCCAGCTT-3’), NLRP1 siRNA2 (5’- GCTTCCAGCATGTCTTCTA-3’), NLRP3 siRNA3 (5’- GCTGGAGCCAAACACCTTT-3’) were purchased from GenePharma (Shanghai, China). U251MG and SHG-44 cells were transfected with siRNA-ctrl, hsa_circ_0001836 siRNA1, hsa_circ_0001836 siRNA2, or hsa_circ_0001836 siRNA3 using Lipofectamine 2000 reagent (Thermo Fisher Scientific) for 48 h. Meanwhile, U251MG cells were transfected with negative control siRNA, NLRP3 siRNA1, NLRP3 siRNA2, or NLRP3 siRNA3 using Lipofectamine 2000 reagent for 48 h.

### RT-qPCR

TRIzol reagent (Takara, Japan) was used to extract total RNA from cells. After that, the RNA was reversely transcribed to cDNA by using an EntiLink™ 1st Strand cDNA Synthesis Kit (ELK Biotechnology, Wuhan, China). The RT reactions were performed as follows: 37˚C for 60 min; 85°C for 5 min. Later on, qPCR was performed using a standard SYBR Premix Ex Taq kit (Takara) on ABI 7500 Real-Time PCR System (Applied Biosystems, Carlsbad, CA, USA). The qPCR reactions were performed as follows: 95°C for 3 min; and 40 cycles at 95°C for 10 s, 58°C for 30 s and 72°C for 30 s. The β-actin gene works as an internal control. The primers were as follows: β-actin, forward, 5’- GTCCACCGCAAATGCTTCTA-3’, reverse, 5’-TGCTGTCACCTTCACCGTTC-3’; hsa_circ_0001836, forward, 5’-GAAGCAGGGGGGTAGAGAGTG-3’, reverse, 5’-TTTTTCCATAGCATTGACAACCA-3’.

### CCK-8 Assay

U251MG and SHG-44 cells (5000 cells per well) were plated onto 96-well plates and incubated overnight at 37°C. After that, the cells were transfected with hsa_circ_0001836 siRNA3 and incubated for 72 h. Then, 10 μl CCK-8 reagent (Sigma Aldrich, St. Louis, MO, USA) was added into each well and incubated for another 2 h at 37°C. Subsequently, the absorbance was measured at 450 nm by using a microplate spectrophotometer (TECAN, Australia).

### EdU Assay

The 5-ethynyl-2′-deoxyuridine (EdU) DNA cell proliferation assay kit (Ribobio, Guangzhou, China) was used to detect the cell proliferation. Briefly, cells were incubated with 50 μM EdU for 2 h, and then fixed in 4% paraformaldehyde, followed by permeabilization with 0.1% Triton-X-100. After that, cells were stained with Apollo dye reagent. Cell nuclei were stained with DAPI for 5 min. Subsequently, the EdU-positive cells were visualized using a fluorescent microscope (Nikon, Japan, Tokyo).

### Flow Cytometry Assay

Cell apoptosis was determined using an Annexin V-FITC/PI Apoptosis detection kit (KeyGen Biotech). U251MG and SHG-44 cells were collected and resuspended in binding buffer. Later on, cells were stained with 5 μl of Annexin V and 5 μl of PI in darkness at 37°C for 30 minutes. After that, cell death rate was analyzed with a FACScan flow cytometer (BD Biosciences, Franklin Lake, NJ, USA) using the CellQuest Pro software (version 5.1). The early-apoptotic cells were Annexin V-positive and PI-negative (Annexin V-FITC^+^/PI^−^), whereas the late-apoptotic/necrotic/pyroptosis cells were Annexin V-positive and PI-positive (Annexin V-FITC^+^/PI^+^).

### Scanning Electron Microscopy (SEM)

The SEM assay was carried out as previously described (17). Cells were harvested and then fixed in ice-cold 2.5% glutaraldehyde for 2 h at room temperature, followed by post-fixation in 1% osmium tetroxide for 1 h. After that, samples were dehydrated in a graded series of ethanol (50, 70, 80, 95 and 100%), and then sputter coated with gold-palladium. Later on, samples were observed using a SEM (Hitachi HT7700, Tokyo, Japan).

### Western Blot Assay

Total protein was extracted from U251MG cells using RIPA buffer for 30 min on ice. The protein concentrations were detected using a BCA protein assay kit (Thermo Fisher Scientific). Total proteins (30 μg per well) were separated on 10% SDS-PAGE and then transferred onto a PVDF membrane. Following blocking with 5% nonfat milk in TBST for 1 h, the membrane was probed with primary antibodies at 4°C overnight. Later on, the membrane was incubated with the corresponding secondary antibodies (1:5000, Abcam Cambridge, MA, USA) for 1 h at room temperature. Subsequently, blots were visualized using enhanced chemiluminescence (ECL) solution (Thermo Fisher Scientific). Primary antibodies used in the assays were NLRP1 (1:1000, Abcam), cleaved caspase 1 (1:1000, Abcam), GSDMD-N (1:1000, Abcam), Pro-caspase 1 (1:1000, Abcam), GSDMD (1:1000, Abcam), and β-actin (1:1000, Abcam).

### ELISA

ELISA kits (ELK Biotechnology, Wuhan, China) were used to determine the production of IL-1β (No. ELK1270) and IL-18 (No. ELK1245) in the supernatant of U251MG cells according to the manufacturer’s protocol.

### Methylation Specific PCR (MSP)

The Genomic DNA Extraction Kit Ver3.0 (Takara, Tokyo, Japan) was used to extract the genomic DNA from U251MG cells. After that, bisulfite conversion was performed by using the EZ-96 DNA Methylation Kit (Zymo Research). The methylated primers of NLRP1 were: 5’- ATTTTAATATTTCGGGAGGTCG-3’ (forward), 5’- ATTACAATCACTCACCACCACG-3’ (reverse); the unmethylated primers of NLRP1 were: 5’-AATTTTAATATTTTGGGAGGTTGA-3’ (forward), 5’- AATTACAATCACTCACCACCACA-3’ (reverse). PCR amplification was conducted at 98°C for 4 min, followed by 40 cycles (98°C for 30 s, 56°C for 30 s, and 72°C for 30 s), and then 72°C for 10 min. Later on, MSP products were analyzed using 3% agarose gel electrophoresis.

### Animal Study

BALB/c nude mice (4-6-weeks old) were obtained from the Shanghai SLAC Animal Center (Shanghai, China). 1 × 10^7^ U251MG cells were injected subcutaneously into the left flank of nude mice. When the tumors reach about 100 mm^3^, animals were randomized into two groups: control, hsa_circ_0001836 siRNA3 group. After that, hsa_circ_0001836 siRNA3 (50 nM) was injected into the tumors directly twice a week. Tumor volume was calculated using the formula: volume = (length × width^2^) x 0.5. After 21 days of treatment, the mice were euthanized, and the entire tumors were isolated and weighed. Tumor tissues were fixed in 10% formaldehyde and subjected to immunohistochemistry (IHC) staining assay. All animal experiments were approved by the Institutional Ethical Committee of the First Affiliated Hospital of Xi’an Jiaotong University, and animals were maintained following the guidelines of the Institutional Animal Care and Use Committee.

### Statistical Analysis

All experiments were repeated three times. All statistical analyses were performed using GraphPad Prism software. One-way analysis of variance (ANOVA) and Tukey’s tests were carried out for multiple group comparisons. Data were expressed as the mean ± standard deviation (S.D.). *P < 0.05 were considered statistically significant.

## Results

### Hsa_circ_0001836 Knockdown Inhibited the Viability and Proliferation of Glioma Cells

To explore the role of hsa_circ_0001836 in glioma cells, we analyzed the level of hsa_circ_0001836 in HA1800 cells, and three glioma cell lines U251 MG, U87MG and SHG-44. According to the results of RT-qPCR, glioma cell (U251 MG and SHG-44) expressed higher hsa_circ_0001836 levels compared to HA1800 cells (**Figure 1A**). Next, we established glioma cell lines (U251 MG and SHG-44) with hsa_circ_0001836 knockdown. Significantly, the level of hsa_circ_0001836 was decreased in U251 MG and SHG-44 cells following transfection with hsa_circ_0001836 siRNA3 (**Figures 1B, C**). In addition, the results of CCK-8 and EdU assays showed that downregulation of hsa_circ_0001836 markedly reduced the viability and proliferation of U251 MG and SHG-44 cells, compared with siRNA-ctrl group (**Figures 1D-F**). Collectively, hsa_circ_0001836 knockdown could suppress the viability and proliferation of glioma cells.

**Figure 1:** Hsa_circ_0001836 knockdown inhibited the viability and proliferation of glioma cells. **(A)** Hsa_circ_0001836 levels in HA1800, U251MG, U87MG and SHG-44 cells were detected using RT-qPCR. **P < 0.01 compared with HA1800 group. **(B, C)** Hsa_circ_0001836 levels in U251MG and SHG-44 cells transfected with hsa_circ_0001836 siRNA1, hsa_circ_0001836 siRNA2 or hsa_circ_0001836 siRNA3 analyzed by RT-qPCR. **(D)** Cell viability analyzed by CCK-8 assay in U251MG and SHG-44 cells transfected with hsa_circ_0001836 siRNA3 for 72 h. **(E, F)** EdU staining assay was used to determine cell proliferation. **P < 0.01 vs. siRNA-ctrl group.

### Downregulation of hsa_circ_0001836 Induced Pyroptosis Cell Death in Glioma Cells

To investigate if the decreases in cell viability after treatment with hsa_circ_0001836 siRNA3 were caused by increased cell death, annexin V/PI analysis was applied. As revealed in **Figures 2A-D**, hsa_circ_0001836 knockdown markedly induced the death of glioma cells. Meanwhile, hsa_circ_0001836 siRNA3 triggered a significant increase of annexin^+^/PI^+^ cells in U251MG and SHG-44 cells when compared with siRNA-ctrl treated cells (**Figures 2A-D**). Since annexin^+^/PI^+^ cells can represent late apoptotic, necrotic and pyroptotic cells, SEM was used to observe the morphology of cells undergoing cell death. As shown in **Figures 2E–F**, U251MG and SHG-44 cells exhibited membrane blebbing, cell swelling and lysis when the cells were transfected with hsa_circ_0001836 siRNA3. Evidences have shown that cells undergoing pyroptosis exhibit cell swelling and lysis and membrane blebbing (18, 19). These data indicated that hsa_circ_0001836 knockdown could trigger the pyroptosis in glioma cells.

**Figure 2:** Downregulation of hsa_circ_0001836 induced pyroptosis cell death in glioma cells. U251MG and SHG-44 cells were transfected with hsa_circ_0001836 siRNA3 for 72 h. **(A–D)** Flow cytometry was used to determine cell death. **(E, F)** Dying cells revealed by SEM. **P < 0.01 vs. siRNA-ctrl group.

### Downregulation of hsa_circ_0001836 Induced Pyroptosis Cell Death in Glioma Cells via Activation of NLRP1-GSDMD Signaling

Pyroptosis is a form of lytic inflammatory cell death triggered by certain inflammasomes, leading to the activation of proinflammatory caspases and the cleavage of gasdermin D (GSDMD) (18, 20). To investigate the mechanism underlying hsa_circ_0001836 siRNA3-regulated pyroptosis in U251MG cells, western blot assay was used. As shown in **Supplementary figure 1A, B**, hsa_circ_0001836 knockdown markedly decreased the expressions of pro-caspase 1 and GSDMD in U251MG cells, compared with siRNA-ctrl group. Meanwhile, downregulation of hsa_circ_0001836 notably upregulated the expressions of NLRP1, cleaved caspase 1 and GSDMD-N in U251MG cells, compared with siRNA-ctrl group (**Figures 3A–D**). In addition, hsa_circ_0001836 knockdown significantly increased IL-1β and IL-18 secretion in U251MG cells (**Figures 3E, F**). These results suggested that hsa_circ_0001836 knockdown could trigger the pyroptosis in glioma cells *via* activation of NLRP1-GSDMD signaling.

**Figure 3:** Downregulation of hsa_circ_0001836 induced pyroptosis in glioma cells *via* activation of NLRP1-GSDMD signaling. U251MG cells were transfected with hsa_circ_0001836 siRNA3 for 72 h. **(A–D)** Western blot analysis of NLRP1, cleaved caspase 1, GSDMD-N levels in U251MG cells. The relative expressions of NLRP1, cleaved caspase 1, GSDMD-N in U251MG cells normalized to β-actin. **(E)** The level of IL-1β in the culture supernatants of U251MG cells was measured using ELISA. **(F)** The level of IL-18 in the culture supernatants of U251MG cells was measured using ELISA. **P < 0.01 vs. siRNA-ctrl group.

### Hsa_circ_0001836 siRNA3 Regulated DNA Methylation of NLRP1 Promoter Region in U251MG Cells

To investigate the molecular mechanism by which hsa_circ_0001836 siRNA3 mediates the upregulation of NLRP1 in U251MG cells, MSP was performed to determine the DNA methylation status of NLRP1 promoter region in U251MG cells. The promoter region of NLRP1 was hypomethylated in hsa_circ_0001836 siRNA3 transfected U251MG cells (**Figure 4A**). These data illustrated that hsa_circ_0001836 siRNA3 could reduce DNA methylation of NLRP1 promoter region in U251MG cells, indicating that hsa_circ_0001836 knockdown may epigenetically increase NLRP1 expression *via* DNA demethylation.

### Downregulation of hsa_circ_0001836 Induced Pyroptosis in Glioma Cells via Epigenetically Upregulating NLRP1

We then we established U251MG cells with NLRP1 knockdown. As indicated in **Figure 4B**, NLRP1 levels were markedly decreased in U251 MG cells following transfection with NLRP1 siRNA2. In addition, CCK-8 assay indicated that inhibitory effects of hsa_circ_0001836 knockdown on cell viability were reversed by the treatment with NLRP1 siRNA2 or a pyroptosis inhibitor necrosulfonamide (NSA) in U251MG cells (**Figure 4C** and **Supplementary figure 2**). Moreover, flow cytometry and SEM assays indicated that downregulation of hsa_circ_0001836 notably induced pyroptosis in U251 cells; however, these changes were reversed by NLRP1 knockdown (**Figures 4D, E**). Meanwhile, hsa_circ_0001836 siRNA3 significantly upregulated the expressions of NLRP1 and GSDMD-N in U251 cells; however, these changes were reversed by NLRP1 siRNA2 (**Figures 4F, G**). Collectively, hsa_circ_0001836 knockdown could trigger the pyroptosis in glioma cells *via* epigenetically upregulating NLRP1.

**Figure 4:** Downregulation of hsa_circ_0001836 induced pyroptosis in glioma cells *via* epigenetically upregulating NLRP1. **(A)** U251MG cells were transfected with hsa_circ_0001836 siRNA3 for 72 h. DNA methylation of the NLRP1 promoter region was analyzed by MSP. “U” and “M” represents unmethylated and methylated signal intensity, respectively. The product length of the methylated primers of NLRP1 is 125 bp; and the product length of the unmethylated primers of NLRP1 is 127 bp. **(B)** The level of NLRP1 in U251MG cells transfected with NLRP1 siRNA1, NLRP1 siRNA2 or NLRP3 siRNA3 analyzed by RT-qPCR. **(C)** U251MG cells were transfected with hsa_circ_0001836 siRNA3 or co-transfected with hsa_circ_0001836 siRNA3 and NLRP1 siRNA2 for 72 h. CCK-8 assay was applied to determine cell viability. **(D)** Cell death was detected by flow cytometry. **(E)** Dying cells revealed by SEM. **(F, G)** Western blot analysis of NLRP1, GSDMD-N levels in U251MG cells. The relative expressions of NLRP1, GSDMD-N in U251MG cells normalized to β-actin. *P < 0.05, **P < 0.01 vs. siRNA-ctrl group; ^##^P < 0.01 vs. hsa_circ_0001836 siRNA3 group.

### Downregulation of hsa_circ_0001836 Inhibited Tumorigenesis in U251MG Xenografts *in Vivo via* Activation of NLRP1-GSDMD Signaling

We next explore the role of hsa_circ_0001836 in regulation of glioma tumor growth *in vivo*. As revealed in **Figures 5A–C**, downregulation of hsa_circ_0001836 significantly reduced the tumor volume and tumor weight, compared with control group. In addition, downregulation of hsa_circ_0001836 markedly decreased the level of hsa_circ_0001836 in tumor tissues (**Figure 5D**). Moreover, hsa_circ_0001836 knockdown notably upregulated the levels of NLRP1, cleaved caspase 1 and GSDMD-N in tumor tissues (**Figures 6A–D**). Meanwhile, IHC analysis indicated that hsa_circ_0001836 knockdown significantly upregulated the levels of IL-1β and IL-18 in tumor tissues of mice (**Figures 6E, F**). These data suggested that knockdown of hsa_circ_0001836 could inhibit tumorigenesis in U251MG xenografts *in vivo via* activation of NLRP1-GSDMD signaling.

**Figure 5:** Knockdown of hsa_circ_0001836 inhibited tumorigenesis in U251MG xenografts *in vivo*. **(A)** Xenograft tumor volume were measured weekly. **(B, C)** Xenografts tumors were imaged on day 21, and the tumor weights were calculated. **(D)** The level of hsa_circ_0001836 in tumor tissues was analyzed by RT-qPCR. **P < 0.01 vs. control group.

**Figure 6:** Knockdown of hsa_circ_0001836 inhibited tumorigenesis in U251MG xenografts *in vivo via* activation of NLRP1-GSDMD signaling. U251 cells (1 × 10^7^ cells) were injected into nude mice subcutaneously, and hsa_circ_0001836 siRNA3 (50 nM) was injected into the tumors directly twice a week. **(A–D)** Western blot analysis of NLRP1, cleaved caspase 1, GSDMD-N levels in tumor tissues. The relative expressions of NLRP1, cleaved caspase 1, GSDMD-N in tumor tissues normalized to β-actin. **(E, F)** IHC analysis was applied to determine the expressions of IL-1β and IL-18 in tumor tissues. **P < 0.01 vs. control group.

## Discussion

CircRNAs have been has been found to play an important role in the progression of glioma (21). In this study, we found that hsa_circ_0001836 is upregulated in glioma cells. Hsa_circ_0001836 knockdown could suppress the viability and proliferation of glioma cells. Meanwhile, hsa_circ_0001836 knockdown could trigger the pyroptosis in glioma cells. Mechanistically, hsa_circ_0001836 knockdown may epigenetically increase NLRP1 expression *via* DNA demethylation, suggesting that hsa_circ_0001836 knockdown could trigger the pyroptosis in glioma cells *via* upregulation of NLRP1.

Pyroptosis, a form of programmed necrosis, is dependent on the activation of caspase-1 (22, 23). Caspase-1 belongs to the group of inflammatory caspases, and can be activated by ligands of various canonical inflammasomes (24). Meanwhile, the activated caspase 1 processes the precursors of IL-1β and IL-18 to the matured IL-1β and IL-18 (25). Besides, the activated caspase 1 can cleave the GSDMD to generate the N-terminal domain (GSDMD-N) (26). The released GSDMD-N can bind to phosphoinositides and then oligomerize in the plasma membrane to generate membrane pores (27). The membrane pores can function as an extracellular gate for release of mature IL-1β and IL-18 (28). In addition, membrane pore formation and membrane disruption can lead to cell swelling and lysis and then pyroptosis (28). In this study, we found that annexin^+^/PI^+^ cells, indicative of late apoptosis, necrosis and pyroptosis, were increased in hsa_circ_0001836 siRNA3 transfected cells. Evidence has shown that the morphology of dying cells can be identified under electron microscopy (22). Our data found that U251MG and SHG-44 cells exhibited membrane blebbing when the cells were transfected with hsa_circ_0001836 siRNA3, whereas cells that undergo necroptosis did not exhibit membrane blebbing (18). Meanwhile, hsa_circ_0001836 siRNA3 led to cell swelling, plasma membrane lysis in U251MG and SHG-44 cells, whereas cells undergoing apoptosis did not exhibit cell swelling and lysis (18). It has been shown that cells undergoing pyroptosis exhibit membrane blebbing, and cell swelling and large bubbles blowing from the plasma (29). Notably, downregulation of hsa_circ_0001836 induced typical pyroptosis in glioma cells, which was elucidated by the bubbles blowing in the membrane and cell swelling. Meanwhile, hsa_circ_0001836 knockdown remarkably upregulated the expressions of NLRP1, cleaved caspase 1 and GSDMD-N in glioma cells both *in vitro* and *in vivo*. These data indicated that hsa_circ_0001836 knockdown could trigger the pyroptosis in glioma cells *in vitro* and *in vivo*.

Evidence has shown that NLRP1 can generate a functional caspase-1-containing inflammasome to trigger pyroptotic death (30, 31). Meanwhile, NLRP1 inflammasome leads to the secretion of IL-1β and IL-18 through the activation of caspase 1 (32). In this study, we found that downregulation of hsa_circ_0001836 notably induced pyroptosis in glioma cells, but that effect was reversed by NLRP1 knockdown. These data suggested downregulation of hsa_circ_0001836 induced pyroptosis cell death in glioma cells *via* upregulation of NLRP1. Interestingly, we found that hsa_circ_0001836 siRNA3 could reduce the methylation levels of NLRP1 promoter region in glioma cells. These data indicated that hsa_circ_0001836 siRNA3 epigenetically increase NLRP1 expression *via* mediating DNA demethylation of NLRP1 promoter region, leading to inhibition of tumor cell growth. Consistently, Liu et al. found that overexpression of circRNA-5692 reduced the methylation levels of the DAB2IP promoter region and increased the expression of DAB2IP in hepatocellular carcinoma (33). We understand that circRNAs have a multitude of remarkable functions, such as microRNA sponge, interaction with RNA binding protein and regulation of gene transcription (34). Xu et al. indicated that lncRNA SATB2-AS1 can bind to WDR5 and GADD45A, cis-activating SATB2 transcription by mediating DNA demethylation of SATB2 promoter region in colorectal cancer cells (35). Chen et al. found that circRNA FECR1 promoted the metastasis of breast cancer *via* inducing DNA demethylation in FLI1 promoter (36). Thus, we are interested in exploring the mechanisms by which hsa_circ_0001836 knockdown decreases the methylation of the NLRP1 promoter region in the glioma.

In recent years, researchers established a U251MG or a SHG-44 *in vivo* model in nude mice to investigate the progression of glioblastoma (37–39). For example, Wang et al. established a U251MG *in vivo* model in nude mice and found that downregulation of circMMP9 markedly inhibited the tumor growth in a xenograft mouse model (37). In this study, we established a U251MG xenograft model, and found that hsa_circ_0001836 knockdown inhibited the tumorigenesis in U251MG xenografts *in vivo via* activation of NLRP1-GSDMD signaling. However, the microenvironment of subcutaneous tumors is different from that of orthotopic tumors (40–42). The immunosuppressive microenvironment has been found to be involved in limiting the efficacy of anticancer drugs (42, 43). Thus, in the future, we plan to establish an intracranial orthotopic glioma model by injection of U251 cells into the left striatum to further investigate the role of hsc-circ-0001836 on the progression of glioma.

## Conclusion

Collectively, we provided the evidence that downregulation of hsa_circ_0001836 inhibited the viability and induced pyroptosis of glioma cells *via* activation of NLRP1-GSDMD signaling. These findings suggested that hsa_circ_0001836 may serve as a potential therapeutic target for the treatment of glioma.

## Data Availability Statement

The original contributions presented in the study are included in the article/**Supplementary Material**. Further inquiries can be directed to the corresponding author.

## Ethics Statement

All animal experiments were approved by the Institutional Ethical Committee of the First Affiliated Hospital of Xi’an Jiaotong University, and animals were maintained following the guidelines of the Institutional Animal Care and Use Committee.

## Author Contributions

QM, YL, and HW designed the project. JJ and HL performed the research. YL and SD collected and analyzed the data. HL and SD analyzed the data. YL wrote the manuscript. QM reviewed and approved the final draft of the manuscript prior to submission. All authors contributed to the article and approved the submitted version.

## Funding

Shanxi National Science Foundation (No. 2019SF-068).

## Conflict of Interest

The authors declare that the research was conducted in the absence of any commercial or financial relationships that could be construed as a potential conflict of interest.

## Supplementary Material

Supplementary Figure 1 Hsa_circ_0001836 knockdown decreased the expressions of pro-caspase 1 and GSDMD in U251 cells. U251MG cells were transfected with hsa_circ_0001836 siRNA3 for 72 h. **(A, B)** Western blot analysis of pro-caspase 1 and GSDMD levels in U251MG cells. The relative expressions of pro-caspase 1 and GSDMD in U251MG cells normalized to β-actin. **P < 0.01 vs. siRNA-ctrl group.

Supplementary Figure 2 Hsa_circ_0001836 knockdown reduced the viability of U251MG cells *via* inducing pyroptosis. U251MG cells were transfected with hsa_circ_0001836 siRNA3 in the absence or presence of 20 μM necrosulfonamide (NSA). CCK-8 assay was applied to determine cell viability. **P < 0.01 vs. siRNA-ctrl group; ^##^P < 0.01 vs. hsa_circ_0001836 siRNA3 group.
